# How Can Different Polishing Timing Influence Methacrylate and Dimethacrylate Bulk Fill Composites? Evaluation of Chemical and Physical Properties

**DOI:** 10.1155/2020/1965818

**Published:** 2020-01-09

**Authors:** Riccardo Monterubbianesi, Vincenzo Tosco, Simona Sabbatini, Giulia Orilisi, Carla Conti, Mutlu Özcan, Giovanna Orsini, Angelo Putignano

**Affiliations:** ^1^Department of Clinical Sciences and Stomatology, Polytechnic University of Marche, Ancona, AN, Italy; ^2^Department of Materials, Environmental Science and Urban Planning, Polytechnic University of Marche, Ancona, AN, Italy; ^3^Dental Materials Unit, Center for Dental and Oral Medicine, Clinic for Fixed and Removable Prosthodontics and Dental Materials Science, University of Zurich, Zurich, Switzerland

## Abstract

The polishing procedure is commonly performed after direct composite restorations, and little information exists regarding the right timing during which it should be performed on bulk fill composites. This study investigated the effect of polishing timing on the degree of conversion (DC), Vickers microhardness (VMH), and surface morphology of a methacrylate- (MET-) and dimethacrylate- (DMET-) based bulk fill composite, by using FT-NIR, microhardness tester, and SEM. Composite samples were divided as follows: in Group I (immediate), samples were polished immediately after curing (*t*_0_); in Group D (delayed), samples were polished after 24 h from curing (*t*_24_), whereas the unpolished samples were considered as controls (Group C). The DC and VMH values were evaluated before and after polishing, at *t*_0_ and *t*_24_. Statistical analysis was performed with a significance level set at *p* < 0.05. At *t*_0_, DC increased after polishing in both tested composites (*p* < 0.05), while at *t*_24_, Group I and Group D were not different. By considering VMH, in the case of MET, all groups were not different both at *t*_0_ and *t*_24_. On the other hand, at *t*_0_, VMH values of DMET increased after polishing. At *t*_24_, DMET Group I and DMET Group D were not different. Qualitative evaluations of scanning electron micrographs showed that the surface morphology of MET presented a more irregular aspect than the DMET one. In summary, since the immediate polishing of MET can improve the DC, without negatively affecting VMH, but showing an irregular surface, it is suggested to wait 24 hours before proceeding with polishing. Otherwise, for DMET, the immediate polishing could definitively be recommended, since it improves both DC and VMH, also producing a regular surface. Therefore, clinicians may always safely polish a restoration performed using DMET-based bulk fill composites in one-chair appointment, avoiding a second appointment.

## 1. Introduction

The light polymerization of dental composites leads to crosslinked networks between monomers inside the resin composites [1]. The formation of these crosslinked networks, evaluated by the degree of conversion (DC), together with the Vickers microhardness (VMH) of materials can have great importance in the success and longevity of dental restorations [2, 3]. It is well known that materials with low DC and VMH enhance the failure rate of reconstruction: a low DC can cause a progressive worsening of the superficial aspect or low biocompatibility, while a low VMH can be linked with low wear resistance and scratches on the reconstruction surface [2, 4]. Moreover, the same DC of different materials can give different VMH [5, 6]. In clinical practice, after the curing of resin composites, clinicians should finish and polish them in order to remove excess of material, fit the occlusion, obtain a smooth surface, and improve their aesthetics [7].

Finishing indicates the contouring or reduction of restoration to obtain ideal anatomy. Polishing reduces the roughness created by finishing [8, 9]. The roughness and an irregular surface lead to plaque accumulation, gingival inflammation, superficial staining, and secondary caries: all of these are some of the frequent reasons for tooth reconstruction failures. Then, an appropriate finishing and polishing are critical clinical procedures that enhance the longevity of restorations [10]. However, polishing and finishing effects depend on the type of resin composites and can influence their chemical and physical properties [11].

In the last few years, the so-called bulk fill composites have been introduced in the market: they consist of a combination of new chemical monomers (methacrylate or dimethacrylate) and fillers with an enhancement of their translucency and, consequently, with the potential of gaining an optimal DC [10, 12]. Although there are many articles on the effects of polishing on traditional resin composites [8, 13], there are no detailed studies concerning the timing effects of the new polishing systems on the properties of bulk fill composites.

Therefore, the aim of this study was to improve the knowledge on these new bulk fill composites, evaluating the effects of immediate and delayed polishing on the DC and VMH of methacrylate and dimethacrylate-based bulk fill composites. The null hypotheses were as follows: (1) the timing of the polishing does not influence the DC of the tested bulk fill composites; (2) the timing of the polishing does not influence their VMH.

## 2. Materials and Methods

The following two bulk fill composites were used: a low-viscosity composite, Estelite Bulk-Fill Flow shade A2 (Tokuyama Dental Inc., Encinitas, CA), which is a methacrylate-based composite (MET), and a high-viscosity composite, Filtek One Bulk Fill Restorative shade A2 (3M, St. Paul, MN, USA), a dimethacrylate-based composite (DMET). Their composition and characteristics are shown in Table 1. For each composite, ten samples were prepared by using homemade Teflon cylinders (3.0 mm in height and 6.0 mm in internal diameter) (Figure 1). All samples were photopolymerized in bulk using Elipar DeepCure S lamp (3M, St. Paul, MN, USA) for 20 sec with an irradiance around 1470 mW/cm^2^ and a spectrum range between 430 and 480 nm. During the photopolymerization, samples were covered with a Mylar strip to exclude oxygen inhibition of surface layer. After curing, the samples were randomly divided into the following groups of five samples for each: MET Group I (I: immediate) and DMET Group I, in which the samples were finished and polished immediately after curing (*t*_0_); MET Group D (D: delayed) and DMET Group D, in which the other samples were finished and polished after 24 h (*t*_24_) from curing. The unpolished samples of Group I at *t*_0_ and Group D at *t*_0_ and *t*_24_ were considered as controls (MET Group C and DMET Group C). Measurements of DC and VMH were performed for all the samples before and after each finishing and polishing procedure, at both *t*_0_ and *t*_24_. Two different disks covered by aluminum oxide (Sof-Lex Disks, 3M, St. Paul, MN, USA) were used to finish the samples: a final contouring medium disk (30 *µ*m abrasive particle size) and a finishing fine disk (14 *µ*m abrasive particle size). The different disk sizes were used in order to simulate the effect of finishing burs which can be used both in anterior and posterior reconstructions. Successively, elastomer wheels impregnated with aluminum oxide and diamond particle (Sof-Lex™ Diamond Polishing System, 3M, St. Paul, MN, USA) were used for the polishing procedures, they consist of a beige prepolishing spiral wheel and a pink high-polishing spiral wheel. Each Sof-Lex disk was used in a circular motion applying light pressure for 10 sec with a slow speed handpiece at 7500 rounds/min. Then, the beige and pink spiral wheels were used with a slow speed handpiece at 6000 rounds/min; a diamond paste (Shiny paste, Enamel Plus, Genova, Italy) was used only with the pink spiral wheel. All the procedures were performed by a single dental operator to minimize operator changes in variability. Each finishing and polishing instrument was discarded immediately after use, and before the evaluations, the samples were washed with distilled water and dried. The samples were stored at 37°C.

### 2.1. Degree of Conversion Analysis

A Perkin Elmer Spectrum One NTS FT-NIR spectrometer equipped with a FR-DTGS detector was used for DC evaluation [5, 14]. For this purpose, on the top of each sample, spectra were acquired in the reflection mode in the 10000–4000 cm^−1^ spectral range, by using the Near Infrared Reflectance Accessory (NIRA) (Perkin Elmer). All the spectra were interpolated, and two-points baseline linear fitted in the 6300–5300 cm^−1^, and the height of the bands at 6165 cm^−1^ and 5990 cm^−1^ was calculated (Spectrum 10.4 software package, Perkin Elmer). The band at 6165 cm^−1^, corresponding to the alkene carbon-carbon double bond vibration (band B), decreased during the polymerization process, while that at 5990 cm^−1^, corresponding to the vibrational modes of the aromatic benzene ring, did not change in intensity (band A). For each spectrum, the ratio between the heights of band B and band A was calculated (band height ratio B/A) [15]. To evaluate the DC, calibration curves were plotted assuming that the ratio B/A of the no cured material may represent the 0% of polymerization, while the same ratio at 1 week, may be taken as 100% of polymerization [5, 16].

### 2.2. Microhardness Analysis

On the same surface of the samples analyzed by FT-NIR spectroscopy, the VMH was determined by using the Leitz microhardness tester (Wetzalr GMBH, Wetzlar, Germany) [14]. The method consisted of indenting the sample by using a pyramid-shaped diamond with a load of 50 g for 15 sec. For each sample, three measurements were performed, respectively, in the middle of the sample, at 0.15 mm and 0.3 mm from the center. After removing the load, the values of the two indentation diagonals were evaluated by using a microscope; the area of the sloping surface was obtained and used to determine the corresponding hardness value. Calculations were made by using Hardness-Course Vickers/Brinell/Rockwell version 10.4.4 software package [17–19].

### 2.3. Surface Evaluation

A Field Emission Scanning Electron Microscope Zeiss Supra 40 (SEM), using a power of 3000 kV and a ×400 magnification, was used for a further surface evaluation of all groups of composites, before and after polishing. The irregularity of the surface was evaluated by using the native software of SEM.

### 2.4. Statistical Analyses of DC and VMH Data

Statistical analysis was performed with R Project for Statistical Computing 3.3.0 (https://www.r-project.org/) and Microsoft Excel 2013. Normality of data distribution and homogeneity of group variances were verified by the Kolmogorov–Smirnov test and the Levene test, respectively. Given the normality and homogeneity of the distribution, one-way analysis of variance (one-way ANOVA) and Tukey's test for comparisons between groups were chosen (*p* < 0.05). The Pearson test was used to evaluate the correlation between the DC and VMH of each material type.

## 3. Results

The statistical evaluations of DC and VMH are reported in Figures 2 and 3, respectively. At *t*_0_, the DC of MET Group C (69.68 ± 3.90) was significantly different from MET Group I (74.88 ± 2.06) (*p*=0.03); at *t*_24_, the difference between the values of all the groups was not significant (MET Group C: 95.53 ± 4.01; MET Group I: 91.73 ± 5.21; MET Group D: 94.21 ± 2.43) (Figure 2(a)). Moreover, all DC MET values of *t*_24_ were different than *t*_0_ values.

On the other hand, at *t*_0_, the DC of the DMET Group C (81.70 ± 2.63) was different from that of DMET Group I (89.57 ± 3.62) (*p*=0.03); at *t*_24_, the difference between the values of all groups was not significant (DMET Group C: 91.78 ± 1.48; DMET Group I: 92.48 ± 4.02; DMET Group D: 91.96 ± 2.62) (Figure 2(b)). Therefore, the DC values of all groups at *t*_24_ were not different from DMET Group I at *t*_0_. However, at *t*_24_, the DC of all polished groups of both composites was not different.

By considering VMH, in MET, both at *t*_0_ and *t*_24_, the difference between the DC values of all groups was not significant (Figure 3(a)). About DMET, at *t*_0_, the VMH values of DMET Group I (88.43 ± 6.17) resulted significantly higher than DMET Group C (81.01 ± 1.01) (*p*=0.02). At *t*_24_, DMET Group I (90.9 ± 3.20) was not significantly different from DMET Group D (85.03 ± 1.98). Moreover, DMET Group I at *t*_24_ was not different from DMET Group I at *t*_0_ (88.43 ± 6.17).

No strong correlation was found between DC and VMH, both in MET (correlation value: 0.16) and DMET (correlation value: 0.40).

SEM results showed that, in the tested materials, different surface patterns may be detected. In MET, the low-viscosity resin composite, both Groups I and D showed an irregular surface (Figures 4(a) and 4(b)). On the other hand, DMET Group I showed a surface smoother and more regular than DMET Group D (Figures 5(a) and 5(b)).

## 4. Discussion

It is well known that the properties of resin composites are material dependent [2, 5, 8]. In clinical practice, considering the oxygen inhibition on the surface, finishing and polishing procedures are important for improving DC and VMH of dental composites, resulting in the success of a restoration [20]. Moreover, finishing and polishing steps are used to modify and improve the profile of a direct composite reconstruction: its success depends on both the type of composite used and the system adopted to finalize it [11, 20]. Although a few reports have investigated the chemical-physical properties of composites after using modern finishing and polishing systems, no studies have evaluated the timing effect of the new polishing system on bulk fill composites containing methacrylate and dimethacrylate monomers [10, 13, 21–23].

In the present study, the Mylar strip was used in order to avoid the oxygen inhibition of the surface layer. DC and VMH of tested composites were evaluated after performing the polishing procedures at different time points. In summary, for DMET the polishing procedure helped the resin composite to reach the same DC recorded at *t*_24_, immediately after curing. On the other hand, for MET, the polishing procedures increase the DC at *t*_0_ even if it did not reach the *t*_24_ values. As hypothesized by the scientific literature, this phenomenon could be explained by the fact that brushing, during polishing, could improve DC due to the heat, generated by the rotary instruments which catalyze the polymerization process on the surface layer [24]. However, the authors speculate that the DC difference between MET and DMET could be based on their monomer combination type: DMET has an addition-fragmentation monomer, which can promote the increase of DC better than methacrylate monomers, during polishing.

Another important property concerning the dental composite and its clinical use is the hardness. It describes the deformation degree of the material, and it is a valuable parameter for making comparison between tooth structure and masticatory forces, especially in the posterior stress-bearing areas [25], thus being considered one of the most important properties. Using materials possessing hardness similar to that of dentin is mandatory to achieve an optimum clinical restoration performance, and this holds mainly for bulk fill composites [26]. Nowadays, clinicians often use bulk fill composites in posterior areas, where their placement is difficult and occlusal forces are more relevant compared to anterior areas [26].

Our results revealed that the hardness of the tested composites, mainly in case of DMET composite, improves after polishing: VMH values of DMET Group I increased after polishing (*p* < 0.05), and they were not statistically different from DMET Group D at *t*_24_ (*p* > 0.05). Regarding VMH of all MET groups, the values were not statistically different (*p* > 0.05). Some authors have hypothesized that, immediately after curing, the surface layer, mostly composed of the organic matrix, may further polymerize during polishing, thus increasing the resistance of the surface layer [13, 27]. However, in our findings, the two tested composites are different not only for the monomers type, but even in vol% and wt%, as well as in filler dimensions. DMET contains a thicker filler (DMET: 4–20 nm versus MET: 200 nm) and a higher wt% and vol% than MET, and consequently, it contains more filler surface to be linked by the matrix monomers and silanes. Maybe, the friction temperature of the polishing procedure could enhance the silanes action [28–30]. The temperature could increase the ability of silanes to link the filler and matrix, improving the hardness. Then, DMET, with a higher filler surface area (more vol% and small filler size), which can link the silanes, could be more influenced by the temperature than MET. Although Chinellatti et al [31] proved that delayed finishing and polishing procedures generally result in a surface similar to or even harder than the one obtained with immediate finishing and polishing procedures, we underline that, in their study, they used flowable, microfilled and minifilled composites, and no bulk fill composites were evaluated. Partially in disagreement with our results, Cenci et al [22] assessed that the polishing procedure, immediately after polymerization, causes incomplete curing and that the stress generated by using rotary instruments may influence the integrity of the restoration, being the range of filler particles a possible explanation for this discrepancy. However, their study dealt only with microfilled or microhybrid resin composites, whereas neither bulk fill composites, specific composite monomers, nor nanofilled composites were evaluated.

In clinical practice, especially in the posterior area, after checking occlusal contacts, clinicians seldom leave composite restorations unfinished and unpolished. It is therefore important to evaluate the occlusal surface of composite materials using various methods, including SEM [32].

The performance of finishing and polishing procedures are often verified using scanning electron micrographs, by qualitatively evaluating shape and contour changes that may not be observed with a profilometer (which gives an objective and quantitative evaluation) [33, 34]. In our study, the characteristics of the tested composites appear different. SEM pictures of both MET groups show more irregular surfaces (>0.2 *μ*m) than DMET ones (Figures 4 and 5), mainly when polishing was performed at *t*_0_.

The formation of an irregular surface on resin composites depends on several material factors, such as the type, shape, size, and distribution of the inorganic filler, and can increase the risk of plaque formation [35–38]. In our case, the presence of thinner filler size results in a reduced matrix interparticle spacing, meaning more protection of the organic matrix and a reduced filler grabbing (as in DMET, with a higher ratio of nanofiller/organic matrix): more organic matrix than filler influences the surface of resin composite because the matrix, less hard than the filler, can show some irregularities after polishing.

Finally, as the previous traditional composites, in both MET and DMET resin composites, no correlation between DC, and VMH was found. It means that not only the DC but also the resin composition influences the mechanical properties of the new bulk fill composites. Although our study presents several limitations, such as the fact that the investigated materials were different in consistency, type of matrix (MET/DMET), and fillers (differently sized particles), it is the first report on the influence of polishing timing on chemical and mechanical properties of the methacrylate- and dimethacrylate-based bulk fill composites.

Therefore, it would be interesting to plan future studies in which other similar high-viscosity bulk fill composites will be analyzed, comparing the correlation among differences in resin monomers and particles content. In particular, the nanotechnological impact of aggregating miscellaneous particles with nanometric dimensions will be taken into account in correlation with the various recently developed monomeric combinations, in order to better understand which is the influence of MET/DMET changes that really improve the clinical performance of these materials.

In summary, the first hypothesis can be rejected. In Group I of both composites, polishing procedures increase the DC at *t*_0_, reaching, mainly in DMET, the same DC of *t*_24_. Furthermore, the second hypothesis can be partially rejected. In the DMET group, the polishing procedure leads to an improvement of VMH, both at *t*_0_ and *t*_24_. Noteworthy is that at *t*_24_, no difference is evident between immediate and delayed polishing of DMET groups. In MET, polishing procedures do not affect VMH values in both groups, whereas DC seems always to be improved.

Our finding may be applied for guiding the clinical use of the above-tested high- (DMET) and low- (MET) viscosity bulk fill composites. In the case of MET, although the immediate polishing improves the DC and VMH is not affected, we recommend waiting 24 hours before polishing, because the surface is more regular in delayed than in immediate polishing. On the other hand, the immediate polishing of restorations performed using DMET could definitively be recommended, since both DC and VMH were increased and a smooth and regular occlusal surface was also observed. Thus, clinicians may always perform and finalize their restorations in one single appointment, saving time, without compromising the good physical properties of these composite resin-based materials.

## Figures and Tables

**Figure 1:** Pictures of homemade Teflon cylinders: frontal (a) and upper (b) view. Height = 3 mm; outside diameter = 10 mm; inside diameter = 6 mm.

**Figure 2:** Degree of conversion values calculated at *t*_0_ and *t*_24_, using different polishing timing for (a) Estelite Bulk-Fill Flow (MET) and (b) Filtek One Bulk Fill (DMET) composites. Tukey test was used, and different superscript letters (A, B, and C) represent statistically significant difference (*p* < 0.05). NP: the samples were not polished; P: the samples were polished; Group I: the samples were cured, finished, and polished immediately after curing; Group D: the samples were cured at *t*_0_ but finished and polished after 24 hours; Group C: the samples were not polished and were used as controls.

**Figure 3:** Vickers microhardness calculated at *t*_0_ and *t*_24_, using different polishing timing for (a) Estelite Bulk-Fill Flow (MET) and (b) Filtek One Bulk Fill (DMET) composites. Tukey test was used, and different superscript letters (A, B, and C) represent statistically significant difference (*p* < 0.05). NP: the samples were not polished; P: the samples were polished; Group I: the samples were cured, finished, and polished immediately after curing; Group D: the samples were cured at *t*_0_ but finished and polished after 24 hours; Group C: the samples were not polished and were used as controls.

**Figure 4:** Scanning electron microscope images (400x magnification) of Estelite Bulk-Fill Flow: (a) MET Group I: polished immediately after curing; (b) MET Group D: polished after 24 hours from curing.

**Figure 5:** Scanning electron microscope images (400x magnification) of Filtek One Bulk Fill Restorative composite: (a) DMET Group I: polished immediately after curing; (b) DMET Group D: polished after 24 hours from curing.

**Table 1:** Composition of the resin-based composites used in this study.

Type	Brand	Composition	Filler load (%)
Bulk fill low-viscosity methacrylate composite	Estelite Bulk-Fill Flow (Tokuyama Dental)	Bis-GMA, Bis-MPEPP, TEGDMA, 200 nm spherical silica, and zirconia SiO_2_–ZrO_2_ 200 nm spherical SiO_2_–ZrO_2_	70.0 wt 56.0 vol

Bulk fill high-viscosity dimethacrylate composite	Filtek™ One Bulk Fill Restorative (3M ESPE)	AFM, AUDMA, UDMA, DDDMA, nonagglomerated/nonaggregated 20 nm silica filler, a nonagglomerated/nonaggregated 4 to 11 nm zirconia filler, an aggregated zirconia/silica cluster filler (comprising 20 nm silica and 4 to 11 nm zirconia particles), and an YbF_3_ filler consisting of agglomerate 100 nm particles	76.5 wt 58.5 vol

w, weight percentage; vol, volume percentage; AFM, addition-fragmentation monomer; AUDMA, aromatic urethane dimethacrylate; Bis-GMA, bisphenol A glycidyl dimethacrylate; Bis-MPEPP, bisphenol A polyethoxy methacrylate; DDDMA 12-dodecane-dimethacrylate; DMA, dimethacrylate; TEGDMA, triethylene glycol dimethacrylate; UDMA, urethane dimethacrylate; YbF3, ytterbium trifluoride.

## Data Availability

The present data used to support the findings of this study are available from the corresponding author upon request.
